# Thermal Ablation of Benign Thyroid Nodules and Papillary Thyroid Microcarcinoma

**DOI:** 10.3389/fonc.2020.580431

**Published:** 2020-10-29

**Authors:** Xiao-Wan Bo, Feng Lu, Hui-Xiong Xu, Li-Ping Sun, Kun Zhang

**Affiliations:** ^1^ Department of Medical Ultrasound, Shanghai Tenth People’s Hospital, Ultrasound Research and Education Institute, Tongji University Cancer Center, Shanghai Engineering Research Center of Ultrasound Diagnosis and Treatment, Tongji University School of Medicine, Shanghai, China; ^2^ Thyroid Institute, Tongji University School of Medicine, Shanghai, China; ^3^ Department of Medical Ultrasound, Shanghai Center for Thyroid Diseases, Shanghai, China

**Keywords:** thyroid nodules, benign thyroid nodules, primary papillary thyroid microcarcinoma, recurrent papillary thyroid microcarcinoma, thermal ablation

## Abstract

Due to the increasing rates of physical examination and application of advanced ultrasound machines, incidences of benign thyroid nodules (BTNs) and papillary thyroid microcarcinoma (PTMC) were dramatically up-regulated in recent years. Thermal ablation (TA) has been widely used and regarded as a safe and effective method to eliminate or reduce BTNs and recurrent low-risk PTMC. However, conclusions using TA to treat primary PTMC are controversial. Recently, several long-term and prospective studies on TA treatment of BTNs and primary PTMC have been reported. Here, we review current literatures and progress on TA treatment of BTNs and PTMC and underline the way to get the best treatment outcomes, providing a comprehensive insight into the research progresses in this field.

## Introduction

Thyroid nodules are frequently detected due to the application of ultrasound examination in recent years (1–5). Most of the nodules are benign thyroid nodules (BTNs) or papillary thyroid microcarcinoma (PTMC). Of note, papillary thyroid carcinoma (PTC) is the most common thyroid cancer but features excellent prognosis and low mortality rate (5, 6). Though active surveillance was recommended for the low-risk PTMC, patients with low-risk PTMC often received aggressive over-treatments (7). Thyroidectomy is the first-line treatment method for BTNs and PTMC according to the 2015 ATA guidelines and 2016 Chinese expert consensus and guidelines (4, 5, 7–9). However, limitations remain unavoidable in reality. On one hand, a few patients may feel fear about or not be appropriate for surgery. On the other hand, thyroidectomy will leave permanent scars and require long-time levothyroxine sodium tablets after surgery, which will cause patients, especially young females, to worry about this treatment. Therefore, alternative minimally surgical techniques or non-surgical invasive treatment methods for thyroid nodules are needed.

Percutaneous chemical ablation (ethanol ablation [EA] or polidocanol injection) was usually used to treat cystic or predominantly cystic BTNs (10–15). Thermal ablation (TA), including radiofrequency ablation (RFA), microwave ablation (MWA), laser ablation (LA), and high intensity focused ultrasound (HIFU), were generally applied for solid or mixed BTNs (15–17). TA therapy for BTNs has been widely utilized across many countries with good efficacy and safety, as revealed by multi-center studies, longitudinal observational studies, guidelines, as well as meta-analyses (18–23). Nevertheless, not all BTNs were appropriate for TA therapy. Long ablation time or multiple ablation operations are needed for the nodules with large sizes. Moreover, fine-needle aspirations (FNA) or core needle biopsy (CNB) was performed to diagnose the thyroid nodules before ablation. However, false negatives may occur in FNA or CNB as they were not the gold standard.

TA was also used for the treatment of recurrent PTMC (24–27). However, the conclusions related to TA of primary PTMC were controversial. Some prospective or retrospective but long-term follow-up studies reported that TA was an effective and safe method for the selected low-risk PTMC (28–30). Before RFA, patients should have no local invasion, regional lymph node, and distant metastasis. Ultrasound and computed tomography (CT) were often used to detect the regional lymph node and distant metastasis (31). However, some regional lymph node metastasis is difficult to detect.

In this present study, we will review the latest progress in TA treatment of BTNs and PTMC to summarize the efficacy and safety of TA techniques, analyze factors related to the efficacy of ablation, and explore future research directions of this topic.

## Patients Included

The selection of patients before TA is related to the safety and efficacy of TA treatment.

### Patients With BTNs

Patients included for TA are as follows: patients with symptomatic or cosmetic problems; patients fearing malignancy; refusal of or contraindications to surgery or radioiodine therapy. The nodules included for TA are as follows: cytological confirmation of a benign thyroid nodule on two separate ultrasound-guided biopsies (ultrasound-guided FNA or CNB); no malignant US findings; solid, predominantly solid, or cystic thyroid nodules; thyrotoxicosis in cases of autonomously functioning thyroid nodules (1, 16, 17, 21–23).

The exclusion criteria are as follows: pregnant women; history of radiation to the neck; follicular neoplasm; severe bleeding tendency because of coagulation disorder; severe heart failure/liver failure/respiratory failure or renal failure; no puncture route judged by US; nodules with heavy calcifications (1, 16, 17, 21–23).

### Patients With PTMC

The inclusion criteria are as follows: refusal of or contraindications to surgery (e.g., age > 80 years or a co-morbidity such as cardiovascular disease, history of stroke, central nervous system vascular malformation, other malignancy, and immunocompromised state); confirmation of PTMC on ultrasound-guided biopsy; no evidence of gross extrathyroidal extension or metastasis (lymphatic or distant metastasis) on both ultrasound and contrast-enhanced computed tomography (CT); either multiple or solitary PTMCs (1, 25–31).

The exclusion criteria are consistent with those patients with BTNs. Moreover, multiple nodules or those PTMCs without ablation safety margin (less than 2 mm away from the thyroid capsule) were also excluded for TA treatment (1, 25–31).

### The Basic Principle of TA

The basic principle of TA is to use the heat energy generated by RF electrode needle, MW antenna, LA fiber, or HIFU to generate coagulative necrosis of the nodules. The coagulation necrotic tissue cells are dissolved and liquefied by hydrolytic enzymes, and they are finally absorbed by lymphocyte and blood vessels. Then the ablation zone gradually decreases and finally disappears completely.

## TA Treatment of BTNs

### RFA

RFA was first reported for the treatment of BTNs in 2006 (32). In the past 10 years, the safety and efficacy of RFA therapy has been validated by some prospective randomized controlled trials (RCTs) and multicenter researches (18–23, 33). The volume reduction rates (VRR) of BTNs were 66.8%–68%, 63%–74.3%, and 70%–82% at 3, 6, and 12 months after RFA, respectively (22, 34–37). Accordingly, therapeutic success (defined as VRR>50%) can be achieved three months after RFA. Intriguingly, some long-term follow-up studies were reported on the efficacy of RFA for BTNs recently (22, 37). For example, a prospective multicenter study indicated that the mean VRR was 80.3%, 84.3%, 89.2%, 91.9%, and 95.3% at 12, 24, 36, 48, and 60 months after RFA treatment (22). Similarly, another retrospective longitudinal observational study reported that the mean VRR was 63%, 67.4%, 66.7%, 66.9%, and 66.9% at the 1-, 2-, 3-, 4-, and 5-year follow-up, respectively (37). Collectively, these long-term follow-up studies showed that VRR remained stable at least one year after RFA.

The symptom and cosmetic problems are the main reasons that patients with BTNs chose to accept treatment. After RFA, patients’ symptom and cosmetic scores were significantly decreased during the follow-up period (22, 34–37). No related deaths were found during and after RFA and the major complication rate was less than 2% (1). Complications such as voice change, pain, hematoma, vomiting, nodule rupture, and Horner syndrome were mostly received after RFA treatment (1). Nevertheless, RFA therapy had fewer complications and pains, preservation of thyroid function as compared with surgery, alongside reduced hospitalization days and increased patients’ satisfaction after RFA (22, 38, 39). Moreover, as patients usually get satisfactory results 3 months after treatment and remain stable at 12 months after RFA, RFA could be considered as the first-line treatment for BTNs for selected patients.

### MWA

Ultrasound-guided percutaneous MWA that was first introduced in 2012 (40) and 2013 in China (41) ranks as the second approach for BTNs treatment. Similar to RFA, MWA is also effective and safe in decreasing the symptom and cosmetic scores for BTNs, even for large (≥3 cm) benign thyroid nodules (18, 42–45). The VRR was 54.3%–75.1%, 68.7%–85.2%, and 88.6%–96.4% at the 3-, 6-, and 12-month follow-up after ablation (17, 42, 44). RFA and MWA showed approximately identical results considering VRR at 3 months follow-up (46). However, RFA showed higher VRRs at the 6- and 12-month follow-up (45). MWA exhibits advanced advantages compared to thyroid lobectomy including faster recovery, fewer complications, more complete thyroid function preservation, superior esthetic results, less physiologic disruption, less expense, and lower systemic stress response (17, 47–49). In summary, MWA should be also considered as one of the first-line treatments for BTNs, especially for larger BTNs since MWA is expected to be more effective based on previous studies. However, more long-term follow-up studies are needed.

### LA

In 2006, ultrasound-guided LA was first introduced for treating patients with BTNs-bearing who are inoperable or unwilling to operate (50). The safety and efficacy of LA of BTNs also have been widely demonstrated, accompanied with significant and persistent volume reduction and local symptom improvement (16, 51–53). The VRR was 55%, 49%–53%, 59%–84% at 3, 6, 12 months follow-up after LA, respectively (51, 54–56). A three-year multicenter prospective randomized trial showed that the VRR was 59%, 60%, and 57% at 1, 2, and 3 years after LA, respectively (56). Compared to RFA and MWA, LA showed similar efficacy and safety considering VRR at 3-months follow-up (56–58). However, the VRR was lower than RFA, but higher than MWA at 6-months follow-up as well as subsequent follow-ups (58–60). From previous literatures, the VRR was relatively low in LA for BTNs. Long-term follow-up studies are also lacking, and more prospective randomized trials are needed to observe efficacy in the future.

### HIFU

HIFU was first reported for the treatment of BTNs in 2011 (61). Subsequently, Lang et al. demonstrated that the mean VRR was 68.87% after 12-month post-HIFU for 22 patients by using nodule volume as the sole determinant of ablation success in a prospective study (62). Lang et al. reported that the mean VRR at 3, 6, 12, 18, and 24 months was 51.32%, 62.99%, 68.66%, 69.76%, and 70.41%, respectively, after HIFU treatment for 108 patients (63). The pooled VRR was 17.59%, 48.93%, and 60.43% at 1, 3, and 6 months after HIFU for BTNs in a systematic review and meta-analysis (64). However, for larger nodules (>20 ml), additional operations were needed at 3–6 months after initial HIFU treatment (65, 66). Compared with open lobectomy, HIFU treatment benefits patients with less treatment time, shortened hospitalization duration, and lower medical cost (67). Noticeably, as a novel and relatively less frequently applied method, HIFU treatment has some drawbacks for the treatment of BTNs, e.g., patients should be stable during HIFU treatment, and longer ablation time and multiple ablation times are needed for patients with large BTNs. Thus, HIFU may be not suitable for patients with large BTNs.

At last, from the long-term retrospective and perspective studies (**Table 1**), RFA showed more effective consequences in reducing nodule volume compared to LA for the treatment of BTNs. Nevertheless, no studies were found on MWA or HIFU for BTNs with more than 2-years follow-up. In addition, few major complications (0%–4.2%) emerged after TA in these long-term follow-up studies (**Table 1**). The most common complications are voice change, vocal cord paresis, laryngeal nerve palsy, intraoperative hemorrhage, and Horner syndrome according to these long-term follow-up studies (**Table 1**). Nevertheless, some nodules regrowth (4.1%–20.4%) after TA still occurred in these studies (**Table 1**). Thus, more prospective and long-term studies are needed in TA treatment of BTNs to obtain the comprehensive conclusions.

**Table 1:** Overview of studies with long-term follow-up on TA treatment of BTNs.

First author/reference no.	Study design	Journal	Country	Case	Method	Nodule volume (ml)	VRR (%) at the 1-, 3-, 6-, 12-, 24-, 36-, 48-, 60-, 72-month	Major complication rate (%)	Regrowth rate (%)
Valcavi (2010) (53)	RCS	Thyroid	Italy	122	LA	23.1 ± 21.3	6.2, NR, 47.5, 50.6, 51.6, 47.8	0	9
Papini (56)	RCT	J Clin Endocrinol Metab	Italy	101	LA	6-17	NR, NR, 49, 59, 60, 57	0.9	NR
Jung (22)	PCS	Korean J Radiol	Korea	345	RFA	14.2 ± 13.2	44.4, NR, NR, 80.3, 84.3, 89.2, 91.9, 95.3	1	NR
Deandrea (37)	RCS	J Clin Endocrinol Metab	Italy	215	RFA	20.9	NR, NR, 56.2, 63, 67.4, 66.7, 66.9, 66.9, 72	0	4.1
Aldea (33)	PCS	J Vasc Interv Radiol	Spain	24	RFA	NR	33.0, 52.1, 56.8, 68.8, 69.9, 76.8,	4.2	NR
Lang (63)	RCS	Eur Radiol	China	136	HIFU	13.09	NR, 51.3, 63.0, 68.7, 70.4	3.7	20.4
Hu (45)	RCS	J Cancer Res Ther	China	100 vs. 72	MWA vs. RFA	13.0 vs. 10.7	24.0, 54.8, 68.7, 75.8 vs. 22.7, 56.1, 77.9, 85.4	4 vs. 2.8	NR

TA, thermal ablation; BTNs, benign thyroid nodules; VRR: volume reduction rates; RCS, retrospective cohort study; PCS, prospective cohort study; RCT, randomized controlled trial; LA, laser ablation; RFA, radiofrequency ablation; HIFU, high intensity focused ultrasound; MWA, microwave ablation; NR, not reported.

## TA Treatment of PTMC

### RFA

RFA could be considered as an alternative method of reoperation objective to recurrent thyroid cancers, as revealed by multiple studies (24–27). For example, Kim et al. reported comparable recurrence-free survival rates between RFA and reoperation for either 1 year (96.0% vs. 92.2%) or 3 year (92.6% vs. 92.2%) groups. The post-treatment complication rates (e.g., hoarseness and hypocalcemia) did not differ significantly between the RFA and reoperation groups (24). In another report, Zhang et al. revealed that the mean VRR was 54%, 81%, 92%, 96%, and 100% at the 1-, 3-, 6-, 12-, and 18-month after RFA, respectively. No residual or recurrent tumor or complications were found during the follow-up period (26). Chung et al. reported that the VRR of RFA for recurrent PTCs was 99.5%, wherein 91.3% of the nodules completely disappeared in the mean 80-months follow-up period (27).

Recently, two studies showed that RFA was also an effective and safe method for primary low-risk PTMC with no local tumor progression or distant metastasis during long-term follow-up (68, 69). As a paradigm, Cho et al. reported that the complete disappearance rates of primary low-risk PTMC were 98.8% and 100% at the 24- and 60-month follow-up after RFA. During the follow-up period, no local tumor progression and lymphatic or distant metastasis were observed. Concurrently, no patients underwent delayed surgery (68). Zhang et al. found that RFA showed similar oncologic outcomes after over 5 years’ follow-up, whereas RFA displayed shorter operation and hospitalization time, lower complications, and less total cost compared with surgery (69). In one study with a large population, 91.4% (139/152) of the ablated low-risk PTMCs completely disappeared with no local or distant recurrence during the mean 39-months follow-up period (31). In terms of health-related life quality, US-guided RFA offers more advantages than surgery, supporting the conclusion that RFA can serve as an alternative strategy for PTMC (70).

### MWA

In 2014, Yue et al. first used ultrasound-guided percutaneous MWA for treatment with PTMC, and in a mean 11-months’ follow-up study, all tumors were completely ablated at a single session and no serious complications occurred (71). Similarly, Teng et al. performed MWA for 21 PTMCs and found that 95.2% of nodules were completely absorbed with no recurrent nodule after 3 years’ follow-up (72). A systematic review and meta-analysis reported that MWA showed significant improvements in nodule volume, clinical symptom scores, and beauty scores between the baseline and final follow-up visits. However, common adverse effects such as hematomas, unbearable pain, and transient or permanent voice change were reported in corresponding 3.8%, 2.2%, and 4.6% of patients from the 33 original articles, but none of these incidents resulted in patients’ hospitalization or death (43). In a 5-year follow-up report, 98.9% of nodules that were diagnosed to be primary PTMC were completely ablated by MWA, with a VRR of 99.37% (30). In a prospective study, 119 unifocal PTMC patients were treated with MWA, VRR was 99.4%, and 93.9% of nodules went into complete remission after mean 37-months follow-up. No residual or recurrent nodules after MWA was observed (29). In a large-cohort study consisting of 185 patients with 206 primary PTMCs, the mean VRR at 21-months follow-up was 98.65% after MWA treatment and 84.5% of nodules were fully absorbed (73). Collectively, these evidences suggest MWA is safe and effective in primary PTMC treatment and offer a new alternative choice for clinical treatment.

### LA

Papini et al. first used LA for local PTMC treatment in an otherwise inoperable patient with thyroid gland at high surgical risk, indicating LA was a safe and effective ablative method (74). Zhou et al. reported that 96.7% (29/30) of the nodules were successfully ablated after a single session. After 1-year follow-up, 33.3% of the ablation zones disappeared, and the remaining 66.67% zones are scar-like nodules. No local recurrence or distant metastases were found in the last follow-up (9). In a retrospective study, the VRR of 81 solitary PTMC treated with LA was 98.4% after mean 49-months follow-up. Compared with surgical group, the patients in the LA group showed shorter hospital stay and procedure time and lower complication and recurrence rates (75). In another retrospective study, 37 patients with primary PTMC were treated with LA, and 32.4% of the treated nodules disappeared and only one patient suffered from cervical lymph node metastasis during 2-years follow-up (76). In summary, LA is also a useful approach for treating primary PTMC.

Interestingly, in the last three years, some long-term follow-up studies summarized that no local recurrence was found after TA of primary PTMC; the recurrence rates in the remaining thyroid were also very low, and few major complications (0%–2.4%) were found during and after the procedure (**Table 2**). The most common complications are voice change and hoarseness (**Table 2**). More than 90% of tumors completely disappeared at the last follow-up period (**Table 2**). However, there are still some nodules requiring additional ablation owing to the insufficient safety margins after the first ablation. In addition, there is no report on the usage of HIFU for the treatment of PTMC yet.

**Table 2:** Overview of studies with long-term follow-up on TA treatment of primary PTMC.

First author/reference no.	Study design	Journal	Country	Method	Case	Follow-up(months)	Complete disappearance rates (%)	Additional ablation (%)	Local recurrence rate (%)	Recurrence in remaining thyroid (%)	LN or distant metastasis rate (%)	Major complications rate (%)
Teng (72)	RCS	J Cancer Res Clin Oncol	China	MWA	21	36	95.2	0	0	0	0	0
Lim (31)	RCS	Korean J Radiol	Korea	RFA	152	39	91.4	9.8	0	0	0	0.8
Zhou (75)	RCS	Int J Hyperthermia	China	LA	36	49	94.4	0	0	0	5.5 (LN)	0
Yue (29)	PCS	J Clin Endocrinol Metab	China	MWA	119	37	93.9	1	0	0	0.8 (LN)	0
Teng (30)	RCS	Thyroid	China	MWA	41	60	97.6	0	0	0	0	2.4
Cho (68)	RCS	Thyroid	Republic of Korea	RFA	84	72	100	15.5	0	4.1	0	1.4
Zhang (69)	RCS	Thyroid	China	RFA	94	64	NR	0	0	1.1	0	0

TA, thermal ablation; PTMC, papillary thyroid microcarcinoma; LN, lymph node; RCS, retrospective cohort study; PCS, prospective cohort study; MWA, microwave ablation; RFA, radiofrequency ablation; LA, laser ablation; NR, not reported.

## Discussion

Eliminating the symptoms or cosmetic problems are the main goals of treating those patients with BTNs. Through systematic and comprehensive reviewing of the field’s progress, we know that all current TA techniques are effective in reducing VRR and patients’ symptoms or cosmetic problems. Fewer complications or adverse events were reported during and after TA for BTNs. Overall, more prospective, multicenter, and long-term follow-up researches were reported in RFA for BTNs than other TA techniques (18, 19, 21–23). Compared with MWA, LA, or HIFU, RFA showed higher VRRs in studies with long-term follow-up for BTNs. Accordingly, RFA may be the preferred treatment for BTNs, and more studies should be carried out on other TA techniques for BTNs.

The symptoms or cosmetic problems are usually found in patients with large nodules. However, the main factors affecting the incomplete ablation were large size and narrow range adjacent to the danger triangle area or carotid artery or trachea and peripheral blood flow (77). Although the overall successful rate is high, the requirement of second-session TA may occur in those cases that nodules are not completed ablated in the first-session treatment. Under such conditions, the total expenses will increase as multiple ablations proceed, which may augment the economic burden of these patients. In addition, as the nodules are not completely ablated, the therapeutic success is difficult to achieve, and the regrowth tends to occur more frequently (78). To avoid these inconveniences, the BTNs should be ablated as completely as possible in one-session treatment.

In addition, factors related to VRR should be critically assessed. The initial volume, initially predominant solidity, clear ill-defined margins, applied energy, and initial ablation ratio were the possible predictive factors of VRR (78–82). For example, over 70% of initial ablation ratio usually predicts VRR of over 50% after RFA (79). However, Lee et al. reported that the VRR of predominantly cystic vs. predominantly solid nodules was similar at 6-months follow-up in a study consisting of 1,000 patients with 1,619 thyroid nodules (78). Moreover, the hardness of the ablation zone after TA may be another factor affecting the VRR despite no association between them reported currently. Collectively, there are no stable predictors of VRR after TA treatment, and more prospective studies on the factors affecting VRR are needed.

The nodule regrowth in BTNs after TA is a critical concern for patients. It is believed that the factors including larger size, the delivery of lower energy, and incomplete and insufficient ablation of the external border of the nodules correlate with regrowth rates (82, 83). Consistent with this, Wang et al. demonstrated that larger initial volume, more irregular blood vessel, and nodules adjacent to the vital structures were found accessible in the recurrence group (84). Recently, Negro et al. suggested that non-spongiform nodules and 12-month VRR < 50% increased the risk of BTNs regrowth after LA in a 5-year follow-up retrospective study (85).

In light of above analysis, the size and location of the nodule are the main factors that affect complete ablation rate, VRR, and nodule regrowth. Regarding this, patients with too large nodules are more suitable for TA. TA can be considered as the first-line treatment for patients with BTNs featuring medium size, even though the symptoms or cosmetic problems are not obvious. However, the specific volume values of larger nodules are uncertain (20, 37, 82). In addition, the new ablation techniques including artery-first ablation, marginal venous ablation, and hydrodissection technique may be useful to decrease the incomplete ablation rate and repress nodule regrowth (86). Thus, it is speculated that more patients will benefit from TA due to the application of advanced ablation techniques.

Interestingly, the successful ablation rates and VRR of TA for PTMC were higher than TA for BTNs during the follow-up periods. Recent long-term prospective and retrospective studies demonstrated that TA was also effective for primary PTMC due to low complications and recurrences (29, 30, 68, 87). From one recent systematic review and meta-analysis, RFA and MWA for primary PTMC were found to show higher VRR than LA (87). Compared with surgery, TAs need less operation and hospitalization time and have a lower total cost. Patients received better health-related life quality, lower total costs, and stress response (69, 70). The major concerns are the lymphatic or distant metastasis in patients with primary PTMC before and after ablation. Actually, low-risk primary PTMCs are rarely found with metastasis, and most metastasis can be found by careful high-resolution ultrasound and CT examination before ablation (7). Moreover, up to now, there have been few researches reporting the local or distant metastasis after TA.

Although patients with low-risk primary PTMC are not recommended for TA treatment, some patients fear metastasis and desire early treatment. Compared with surgery, patients benefit from TA, typically associating with shorter treatment and hospitalization time, lower complications, and no neck scars. Moreover, RFA, MWA, or LA showed similar efficacy and safety on the basis of previous long-term follow-up studies. Taken together, TA is a promising alternative treatment for patients with low-risk primary PTMC.

Although TA is an effective and safe method for the treatment of BTNs and low-risk primary PTMC, some limitations of TA should also receive more attention. First, TA is not suitable for all types of thyroid nodules comparing with surgery, especially for large BTNs, substernal nodules, and deep located nodules. Second, there are still some nodules with incomplete response and local regrowth in the following-up period, which will need repeated ablation or surgery. Third, some nodules shrunk slowly but failed to completely recede according to the current studies. Accordingly, more studies focusing on improving the effectiveness of ablation and reducing local or distant recurrence of nodules are demanded in the future.

### Outlook

In this review, some prospective and prospective clinical studies with long follow-up periods showed that TA was effective and safe for the treatment of BTNs and PTMC. Nevertheless, more prospective randomized controlled trials of large samples comparing TA with surgery with more than five-year follow-up are still absent. Moreover, it is also unsure on whether TA is also effective for the treatment of large PTC or other pathological subtypes of thyroid carcinoma. In addition, the dissolved gas will give birth to bubbles that usually cause strong backscattering ultrasonic signals, which inevitably introduces mistakes into the assessment and monitoring of the ablation process and lesion boundary. To overcome this issue, new imaging technology featuring precise ablation guidance and curative assessment will also be explored. Intriguingly, some fundamental researches on enhancing thermal sensitivity using some enhancement agents were highlighted to improve the utilization efficiency of thermal energy, elevate treatment biosafety, and magnify the ablation outcomes. These impressive cases pave a solid foundation to clinical translation of these enhancement agents *via* providing theoretical basis and experimental experiences, e.g., RFA enhancement agents, HIFU enhancement agents, etc.

## Conclusions

Thermal ablation is a promising minimally invasive method and should be considered as the first-line treatment for BTNs and recurrent PTMC. For primary PTMC, TA could be a suitable alternative to surgery for selected patients with low-risk PTMC. However, the suitable included criterion, the ablation equipment selection, and the standard technical operation should be critically evaluated to ensure the best clinical outcomes and complication control after ablation.

## Author Contributions

All authors: designed and wrote the manuscript. X-WB, FL: drafted the manuscript and prepared the tables. L-PS, KZ, and H-XX: modified the manuscript. All authors contributed to the article and approved the submitted version.

## Funding

This work was supported by grants from National Natural Science Foundation of China (Grants 82022033, 81771836, 81501473, 81601501 and 81801802), Shanghai Rising-Star Program (Grant 19QA1406800), Shanghai Talent Development Fund (Grant2019040), Fostering Project of Shanghai Municipal Commission of Health and Family Planning for Excellent Young Medical Scholars (Grant 2018YQ31), the Opening Project of Guangxi Key Laboratory of Bio-targeting Theranostics (GXSWBX201801), the Opening Project of State Key Laboratory of High Performance Ceramics and Superfine Microstructure (SKL201811SIC), Shanghai Municipal Health Commission (Grant201640166), and Shanghai “Rising Stars of Medical Talent” Youth Development Program.

## Conflict of Interest

The authors declare that the research was conducted in the absence of any commercial or financial relationships that could be construed as a potential conflict of interest.
